# Diagnostic Value of Image Features of Magnetic Resonance Imaging in Intracranial Hemorrhage and Cerebral Infarction

**DOI:** 10.1155/2022/6495568

**Published:** 2022-07-12

**Authors:** Wencai Tang, Fangyi Zeng, Guangtang Zhao

**Affiliations:** ^1^Department of Radiology, The Second Affiliated Hospital of Hainan Medical University, Haikou 570000, Hainan, China; ^2^Department of Radiology, Hainan Danzhou People's Hospital, Danzhou 571700, Hainan, China

## Abstract

This study aimed to investigate the differential diagnosis value of routine magnetic resonance imaging (MRI) and magnetic resonance diffusion-weighted imaging (DWI) in hyperacute intracranial hemorrhage (HICH) and hyperacute cerebral infarction (HCI). Fifty-five patients with HICH were set as group A, and 55 patients with HCI were selected as group B. All the patients underwent routine MRI and DWI examinations. The morphological distribution and signal characteristics (low, high, or mixed) of the lesions in the two groups were recorded. The diagnostic accuracy, sensitivity, and specificity of routine MRI and DWI were compared for distinguishing HICH and HCI. The results suggested that the lesions in patients with HICH were mainly manifested as mixed signals (40 cases), while those in patients with HCI showed high signals (48 cases). HICH occurred in the basal ganglia in 44 cases, in the brain stem in 6 cases, in the cerebellum in 4 cases, in the cerebral cortex in 0 cases, and in the corpus callosum in 1 case. HCI occurred in the basal ganglia area, brain stem, cerebellum, cerebral cortex, and corpus callosum in 5, 3, 35, 12, and 0 cases, respectively. The diagnostic accuracy, specificity, and sensitivity of DWI for HICH and HCI were significantly higher than those of routine MRI (*P* < 0.05). It was indicated that compared with routine MRI, DWI was more effective in the diagnosis of HICH and HCI, with clearer and more accurate images and better diagnostic performance.

## 1. Introduction

Stroke, also known as a cerebrovascular accident, is an acute cerebrovascular disease. It is a group of diseases that cause brain tissue damage due to sudden rupture of blood vessels in the brain or the inability of blood to flow into the brain due to vascular obstruction, including ischemic and hemorrhagic stroke [1–3]. Statistically, the incidence of ischemic stroke is higher than that of hemorrhagic stroke, accounting for about 65% of all strokes [4, 5]. Stroke occurs in people more than 40 years old, more men than women; in severe cases, it can cause death. Stroke can also be divided into intracranial hemorrhage and cerebral infarction, of which cerebral infarction is caused by cerebral thrombosis, atherosclerosis, cardioembolic embolism, etc. These result in the sudden interruption of blood flow in the cerebral blood vessels, causing local brain tissue necrosis and thereby forming symptoms of neurological deficits. Intracerebral hemorrhage is caused by the spontaneous rupture and hemorrhage of cerebral blood vessels, which causes the blood in vessels to overflow into the parenchymal cells of the brain, resulting in necrosis and swelling of the patient's brain tissue [6, 7]. Clinically, intracerebral hemorrhage and cerebral infarction that occur within 6 hours are called hyperacute intracranial hemorrhage (HICH) and hyperacute cerebral infarction (HCI). However, there are obvious differences between the two, and the treatment options are also completely different [8]. Therefore, the accurate identification of HICH and HCI within 3–6 hours of onset has a great influence on the effectiveness of treatment for patients.

In recent years, with the rapid development of medical imaging technology, various imaging methods can not only indicate morphological changes in brain tissue but also provide information on cerebral blood flow and metabolism, playing an important role in early diagnosis and treatment [9–12]. Computerized tomography (CT) utilizes precise and accurate X-ray beams, gamma rays, ultrasonic waves, etc., together with highly sensitive detectors, to scan a certain part of the human body one plane by one plane. It has the characteristics of fast scanning and clear images. It is often used in the clinical diagnosis of stroke, but with low sensitivity [13, 14]. Magnetic resonance imaging (MRI) can map the internal structure of an object according to the different attenuation of the released energy in different structural environments inside the material as well as the emitted electromagnetic waves detected in a gradient magnetic field. Taking advantage of the high resolution, multi-parameters, and so on, it has also been gradually applied to the clinical diagnosis of stroke, but there are certain limitations as well [15–17]. Diffusion-weighted imaging (DWI), as a new MRI method, is different from traditional T1-weighted imaging (T1WI) and T2-weighted imaging (T2WI). It can describe the diffusion process of molecules (especially water molecules) in biological tissues through specific MRI sequences and software to generate images from the resulting data [18, 19]. At present, most of the studies on the diagnosis by DWI are aimed at the symptoms of cerebral infarction, and the diagnostic effect of cerebral hemorrhage is not completely clear.

To sum up, imaging techniques are common to diagnose stroke, but there are differences in the application effects of various imaging techniques to a certain extent. It is necessary to choose the most reliable examination method. Thus, 55 patients with HICH were included in group A, while 55 patients with HCI were included in group B. Routine MRI and DWI examinations were performed on all the patients, and the pathological diagnosis results were used as the gold standards. The diagnostic accuracy, sensitivity, and specificity of routine MRI and DWI for HICH and HCI were calculated to innovatively explore the diagnostic performance of different MRI imaging techniques for HICH and HCI.

## 2. Materials and Methods

### 2.1. Research Objects

Fifty-five patients with HICH and 55 patients with HCI were chosen as the research objects, as they were admitted to the hospital from October 2020 to December 2021. The 55 cases with HICH were included in group A, and the 55 cases with HCI were in group B. This study had been approved by the ethics committee of the hospital, and all patients participated voluntarily and signed informed consent forms.

Inclusion criteria: if the patients could offer complete basic information, had no contraindications to MRI examination, signed the informed consent, and were older than 20 years old.

Exclusion criteria: if the patients were complicated with mental illness, complicated with heart, liver, and kidney dysfunction, or complicated with diseases of the blood system. Patients had poor compliance in examinations, or they withdrew from the project due to personal reasons.

### 2.2. Imaging Methods

The patients were examined with a fiber-optic superconducting 1.5 T magnetic resonance instrument. Scanning parameters for routine MRI and DWI (coronal T1WI, coronal T2WI, and fluid-attenuated inversion recovery (FLAIR)) are listed in Table 1.

### 2.3. Image Processing

The obtained images under routine MRI and DWI were read by two senior radiologists using a double-blind method. After the image data were sent to the General Electric workstation, the hematoma or infarction locations were selected in the original window for image correction. The apparent diffusion coefficient (ADC) maps were obtained after processing, and the ADC values of the lesions of HICH and HCI were measured. With 0.8 × 10^−3^ mm^2^ taken as the boundary, there were two intervals of 0.4–0.8 × 10^−3^ mm^2^ and 0.8–1.2 × 10^−3^ mm^2^.

### 2.4. Observation Indicators

The general data of the patients (male to female ratio, average age, average height, average weight, proportion of high blood pressure, proportion of diabetes, and proportion of smoking history) were recorded. The images of patients with HICH and HCI were compared, and the morphological distribution and the low, high, or mixed signal characteristics of the lesions were also recorded. The diagnostic accuracy, sensitivity, and specificity of routine MRI and DWI for HICH and HCI were calculated with pathological diagnosis results as the gold standards. The ADC values of patients with HICH and HCI were compared as well.

### 2.5. Statistical Methods

The SPSS 19.0 statistical software was used for data processing. Measurement data were expressed as mean ± standard deviation (±*S*), while enumeration data were expressed as percentage (%). One-way analysis of variance was adopted for the pairwise comparisons of the indicators of patients between group A and group B. The difference was statistically significant at *P* < 0.05.

## 3. Results

### 3.1. Comparison of General Data

Figure 1 showed the comparison of the patients' general data between the two groups. The ratio of male to female, the average age, the average height, the average weight, the proportion of high blood pressure, the proportion of diabetes, and the proportion of smoking history in group A were all not significantly different from those in group B (*P* > 0.05).

### 3.2. Imaging of Patients with HICH and HCI

Figure 2 displays the images of a patient with HICH. There was oxygenated hemoglobin in the right lateral ventricle, which had a slight effect on the MRI signal. T1WI showed a low signal, T2WI showed a high signal, but the T2WI signal was uneven. The images of a patient with HCI were presented in Figure 3. The lesion was shown with an obvious high signal, together with the strip-shaped high signal shadow inside.

### 3.3. Signal Comparison of Lesions

In Figure 4, the signals of the lesions in patients were compared between the two groups. The lesions in patients with HICH were dominated by mixed signals. 40 cases were shown under DWI (72.73%) and 21 cases were under routine MRI (38.18%); the difference was considered to be statistically significant (*P* < 0.05). The lesions in patients with HCI were mainly shown as high signals, among which 48 cases were shown under DWI, accounting for 87.27%. 30 cases were shown by routine MRI, which accounted for 54.55%, and the difference was also of statistical significance (*P* < 0.05).

### 3.4. Comparison of ADC Values

The ADC values of the two groups of patients were compared in Figure 5. There were 12 patients in group A whose ADC value was in the range of 0.4–0.8 × 10^−3^ mm^2^, and 43 patients whose ADC value was 0.8–1.2 × 10^−3^ mm^2^. In group B, the ADC value of 0.4–0.8 × 10^−3^ mm^2^ was found in 43 cases and that of 0.8–1.2 × 10^−3^ mm^2^ was found in 16 cases. There was a statistically significant difference in ADC value between group A and group B (*P* < 0.05).

### 3.5. Comparison of Imaging Examination Performance

Figure 6 displays the comparison of the diagnostic accuracy, sensitivity, and specificity between the two groups as well as between routine MRI and DWI. For diagnosing HICH by routine MRI, the accuracy was 73.12%, the sensitivity was 79.66%, and the specificity was 65.37%. The diagnostic accuracy, sensitivity, and specificity of DWI were 96.33%, 92.65%, and 85.15%, respectively. For HCI, the diagnostic accuracy of routine MRI was 65.81%, the diagnostic sensitivity was 81.45%, and the diagnostic specificity was 70.32%. The diagnostic accuracy, sensitivity, and specificity of DWI for HCI were 97.14%, 90.74%, and 82.45%, respectively. The accuracy, specificity, and sensitivity of DWI for diagnosing both HICH and HCI were significantly higher than those of routine MRI, showing statistically significant differences (*P* < 0.05).

### 3.6. Comparison of the Lesion Locations in the DWI Examination

Figure 7 shows the comparison of lesion locations in the two groups in the DWI examination. In DWI examination, HICH occurred in the basal ganglia, brain stem, cerebellum, cerebral cortex, and corpus callosum in 44, 6, 4, 0, and 1 cases, respectively. HCI occurred in those locations in 5 cases, 3 cases, 35 cases, 12 cases, and 0 cases, respectively.

## 4. Discussion

Stroke is a common clinical disorder of cerebral blood circulation, generally divided into cerebral infarction and intracerebral hemorrhage. If the diseases occur within 6 hours, it is called the hyperacute phase [20, 21]. Clinically, the optimal treatment time for stroke is 3–6 hours, in which the best prognosis can be achieved for patients. However, because the clinical manifestations of cerebral infarction and intracerebral hemorrhage are similar, the treatment options are different. It is necessary to seek an efficient and high-precision method to distinguish HICH from HCI [22]. The commonly used clinical examination methods are CT and MRI techniques, but the diagnostic sensitivity of both CT and routine MRI is not high. It is prone to missing and misdiagnosing some cases, which will lead to delay and aggravation of the patients' condition [23, 24]. Different from the traditional MRI technology, DWI can use the pulse sequence sensitive to the diffusion movement to detect the diffusion motion state of water molecules in the tissue and then express it in MRI images. Therefore, 55 patients with HICH and 55 patients with HCI, admitted to the hospital from October 2020 to December 2021, were included as the research objects. The patients with HICH and HCI were in group A and group B, respectively, and all of them experienced routine MRI and DWI examinations. First, the general data of the patients in two groups were compared, and it was known that the ratio of males to females, the average age, the average height, the average weight, the proportion of high blood pressure, the proportion of diabetes, and the proportion of smoking history in group A were not remarkably different from those in group B (*P* > 0.05). Such a result provided a feasibility for subsequent analyses, and the results would be reliable [25].

From the images, the oxygenated hemoglobin was observed in the right lateral ventricle of patients with HICH. The low signal was shown on T1WI and the high signal on T2WI, but the signal on T2WI was uneven. The lesion in HCI patients showed obvious high signal with strip-shaped high signal shadow insides. It was indicated that the signal levels of HICH and HCI were different in MRI images [26, 27]. The quantitative data showed that the lesions in patients with HICH were dominated by mixed signals (40 cases), while those in patients with HCI were dominated by high signals (48 cases). These were consistent with what the above images presented, further confirming that there were significant differences in the signal of lesions. In terms of lesion location, 44 HICH cases had their lesion in the basal ganglia, 6 cases in the brain stem, 4 cases in the cerebellum, 0 cases in the cerebral cortex, and 1 case in the corpus callosum. There were 5, 3, 35, 12, and 0 HCI cases that had lesions in the basal ganglia, the brain stem, the cerebellum, the cerebral cortex, and the corpus callosum, respectively. Thus, it could be concluded that HICH mostly occurred in the basal ganglia region, while HCI occurred in the cerebellum and cerebral cortex mostly, showing the very distinct difference between the two [28].

In addition, the performances of routine MRI and DWI were also compared in the detection of HICH and HCI. For HICH, there were 40 cases of mixed signal under DWI, accounting for 72.73%; and 21 cases of mixed signal under MRI, accounting for 38.18%. The difference was statistically significant (*P* < 0.05). For HCI, 48 cases were observed with high signal under DWI (87.27%), 30 cases with high signal under MRI (54.55%), and the difference was of statistical significance (*P* < 0.05). These indicated that DWI images had a significant effect on the clearer and more accurate display of HICH and HCI, showing a high signal of HCI and a mixed signal of HICH. DWI had a high reference significance for the differential diagnosis of the two diseases. The diagnostic accuracy, specificity, and sensitivity of DWI for HICH and HCI were significantly higher than those of routine MRI, with differences of statistical significance (*P* < 0.05). This was similar to the findings of Zhao et al. [29], suggesting that DWI could better show the functional and physiological changes of water molecules in human tissues. Therefore, DWI was superior to routine MRI in the detection of both the diseases.

## 5. Conclusion

The diagnostic value of routine MRI and DWI was discussed in 55 patients with HICH and 55 patients with HCI. The lesions in patients with HICH showed mixed signals mainly, which were mostly in the basal ganglia. The lesions in patients with HCI were represented by high signals and were mostly in the cerebellum and cerebral cortex. DWI produced clearer and more accurate images than routine MRI for the display of HICH and HCI, showing high-signal characteristics of HCI and mixed-signal characteristics of HICH. The diagnostic accuracy, sensitivity, and specificity of DWI were also higher. However, there were still some unresolved issues in this research. The sample size of the patients included was small and the source was single, and there was also a lack of long-term data on the prognosis of patients. The impact of the DWI examination on the prognosis of patients was not discussed. The patient samples would be re-included in the future for a deeper analysis. In conclusion, the results provided data reference for the imaging differentiation of HICH and HCI.

## Figures and Tables

**Figure 1:** Comparison of the general data of patients in the two groups. (a) The comparison of gender; (b) age, height, and weight comparison; (c) proportion of high blood pressure, diabetes, and smoking history comparison.

**Figure 2:** Imaging data of a patient with HICH. (a–e): T1WI, T2WI, pressurized-water T2WI, DWI, and FLAIR, respectively.

**Figure 3:** Imaging data of a patient with HCI. (a–e): T1WI, T2WI, pressurized-water T2WI, DWI, and FLAIR, respectively.

**Figure 4:** Comparison of the signals of the lesions in the two groups of patients. (a–c) showed the comparison of low signal, high signal, and mixed signal, respectively. ^*∗*^Compared with the corresponding signal under DWI, *P* < 0.05; ^#^compared with that in group B *P* < 0.05.

**Figure 5:** Comparison of ADC values between the two groups of patients. 1 stood for 0.4–0.8 × 10^−3^ mm^2^, and 2 meant 0.8–1.2 × 10^−3^ mm^2^. ^*∗*^Compared with the data of group A *P* < 0.05.

**Figure 6:** Comparison of the diagnostic accuracy, sensitivity, and specificity of the two groups by routine MRI and DWI. (a) Comparison of the accuracy; (b) the sensitivity; (c) the specificity. ^*∗*^Compared with the data under DWI, *P* < 0.05.

**Figure 7:** Comparison of lesion locations in the DWI examination between two groups. 1–5 represented the basal ganglia, brainstem, cerebellum, cerebral cortex, and corpus callosum, respectively.

**Table 1:** Imaging scan parameters.

Parameters	Routine MRI	T_2_WI	T_1_WI	FLAIR
Slice thickness	1.5 mm	5 mm	1.2 mm	1.2 mm
Slice spacing	5 mm	1.5 mm	4 mm	4 mm
Matrix	256 × 256	256 × 185	256 × 185	256 × 185
Field of view	150 × 220 mm	220 × 220 mm	220 × 220 mm	220 × 220 mm
Time of echo/time of repetition	580 ms/35 ms	660 ms/40 ms	660 ms/40 ms	660 ms/40 ms

## Data Availability

The data used to support the findings of this study are available from the corresponding author upon request.

## References

[1] Kimura H. (2020). Stroke. *Brain and Nerve*.

[2] El-Koussy M., Schroth G., Brekenfeld C., Arnold M. (2014). Imaging of acute ischemic stroke. *European Neurology*.

[3] Knight-Greenfield A., Nario N., Gupta A. (2019). Causes of acute stroke. *Radiologic Clinics of North America*.

[4] de Mendivil A. O., Alcalá-Galiano A., Ochoa M., Salvador E., Millán J. M. (2013). Brainstem stroke: anatomy, clinical and radiological findings. *Seminars in Ultrasound, CT and MRI*.

[5] Bersano A., Kraemer M., Burlina A. (2021). Heritable and non-heritable uncommon causes of stroke. *Journal of Neurology*.

[6] Simonsen C. Z., Leslie-Mazwi T. M., Thomalla G. (2021 Jan). Which imaging approach should Be used for stroke of unknown time of onset. *Stroke*.

[7] Murray N. M., Unberath M., Hager G. D., Hui F. K. (2020 Feb). Artificial intelligence to diagnose ischemic stroke and identify large vessel occlusions: a systematic review. *Journal of Neurointerventional Surgery*.

[8] Sparaco M., Ciolli L., Zini A. (2019). Posterior circulation ischemic stroke-a review part II: imaging and acute treatment. *Neurological Sciences*.

[9] Suri R., Rodriguez-Porcel F., Donohue K. (2018 Sep). Post-stroke movement disorders: the clinical, neuroanatomic, and demographic portrait of 284 published cases. *Journal of Stroke and Cerebrovascular Diseases*.

[10] Lv Z., Qiao L., Wang Q., Piccialli F. (2021). Advanced machine-learning methods for brain-computer interfacing. *IEEE/ACM Transactions on Computational Biology and Bioinformatics*.

[11] Inatomi Y., Nakajima M., Yonehara T., Ando Y. (2017). Ipsilateral hemiparesis in ischemic stroke patients. *Acta Neurologica Scandinavica*.

[12] Yu Z. C., Amin S. U., Alhussein M., Lv Z. H. (2021). Research on disease prediction based on improved DeepFM and IoMT. *IEEE Access*.

[13] Hu M., Zhong Y., Xie S., Lv H., Lv Z. (2021). Fuzzy system based medical image processing for brain disease prediction. *Frontiers in Neuroscience*.

[14] Amatangelo M. P. (2020). Cryptogenic stroke. *Critical Care Nursing Clinics of North America*.

[15] Ferrara A. (2020). Computed tomography in stroke diagnosis, assessment, and treatment. *Radiologic Technology*.

[16] Xie S. X., Yu Z. C., Lv Z. H. (2021). Multi-Disease prediction based on deep learning: a survey. *Computer Modeling in Engineering and Sciences*.

[17] Dolotova D., Donitova V., Arhipov I. (2019). A platform for collection and analysis of image data on stroke. *Studies in Health Technology and Informatics*.

[18] Hart R. G., Diener H. C., Coutts S. B. (2014). Embolic strokes of undetermined source: the case for a new clinical construct. *The Lancet Neurology*.

[19] Wang G., Song T., Dong Q., Cui M., Huang N., Zhang S. (2020). Automatic ischemic stroke lesion segmentation from computed tomography perfusion images by image synthesis and attention-based deep neural networks. *Medical Image Analysis*.

[20] Yang R., Zhang Y., Xu M., Ma J. (2021). Image features of magnetic resonance angiography under deep learning in exploring the effect of comprehensive rehabilitation nursing on the neurological function recovery of patients with acute stroke. *Contrast Media and Molecular Imaging*.

[21] D’Anna L., Filippidis F. T., Harvey K., Korompoki E., Veltkamp R. (2022). Ischemic stroke in oral anticoagulated patients with atrial fibrillation. *Acta Neurologica Scandinavica*.

[22] Kitsiou A., Zuhorn F., Wachter R., Israel C. W., Schäbitz W. R., Rogalewski A. (2021). Embolischer Schlaganfall mit ungeklärter Emboliequelle (ESUS) - klassifikation einer neuen Schlaganfallentität. *DMW - Deutsche Medizinische Wochenschrift*.

[23] Nutakki A., Chomba M., Chishimba L. (2021). Risk factors and outcomes of hospitalized stroke patients in Lusaka, Zambia. *Journal of the Neurological Sciences*.

[24] Bates V. (2009). Outpatient neuroimaging of stroke. *Neurologic Clinics*.

[25] Ayrignac X., Gaillard N., Carra-Dallière C., Labauge P. (2020). Microangiopathie cérébrale: du diagnostic à la prise en charge small vessel disease of the brain: diagnosis and management. *La Revue de Medecine Interne*.

[26] Boustia F., Crespy A., Janot K., Herbreteau D. (2019). Prise en charge endovasculaire de l’accident vasculaire cérébral ischémique aigu. *La Presse Médicale*.

[27] Yu A. Y. X., Hill M. D., Coutts S. B. (2015). Should minor stroke patients be thrombolyzed? A focused review and future directions. *International Journal of Stroke*.

[28] Bao L., Zhang S., Gong X., Cui G. (2020). Trousseau syndrome related cerebral infarction: clinical manifestations, laboratory findings and radiological features. *Journal of Stroke and Cerebrovascular Diseases*.

[29] Zhao D., Zhu J., Cai Q., Zeng F., Fu X., Hu K. (2022). The value of diffusion weighted imaging-alberta stroke program early CT score in predicting stroke-associated pneumonia in patients with acute cerebral infarction: a retrospective study. *PeerJ*.

